RETRACTED

# LINC00337 Regulates KLF5 and Maintains Stem-Cell Like Traits of Cervical Cancer Cells by Modulating miR-145

**DOI:** 10.3389/fonc.2020.01433

**Published:** 2020-08-14

**Authors:** Qi Han, Wenjin Wu, Yulan Cui

**Affiliations:** Department of Obstetrics and Gynecology, The Second Affiliated Hospital of Harbin Medical University, Harbin, China

**Keywords:** cervical cancer, cancer stem-like cells, long non-coding RNA, LINC00337, microRNA-145, Kruppel-like factor 5

## Abstract

Accumulating literature and evidence has highlighted the cancer stem-like cell (CSC) model as a cellular mechanism responsible for the phenotypic heterogeneity observed in various types of cancers, including cervical cancer. Long non-coding RNAs (lncRNAs) have been implicated in the retention of stem cell-like traits in cancer cells. However, the role of lncRNAs in the acquisition and maintenance of CSCs in cervical cancer remains largely unknown. Hence, the current study identified that LINC00337 knockdown diminished the CSC-like properties of CD44^+^/CD24^low/−^SFCs, evidenced by a decline in the generation of tumorospheres and colonies, a reduction in multi-drug resistance gene-1 (MDR-1), Nanog, Sox2, and Oct4 expression, along with an enhancement in cell apoptosis. RNA pull-down assays and RNA immunoprecipitation revealed the role of LINC00337 as a competing endogenous RNA (ceRNA) of microRNA-145 (miR-145). Furthermore, the miR-145 mRNA target, Kruppel-like factor 5 (KLF5), was decreased in CD44^+^/CD24^low/−^SFCs upon LINC00337 knockdown. The *in vitro* results were reproduced in *in vivo* studies, which provided verification attesting that LINC00337 knockdown attenuated the tumorigenicity of CD44^+^/CD24^low/−^SFCs in nude mice. Taken together, the key findings of the current study demonstrate that LINC00337 acts as an oncogenic lncRNA in cervical cancer and exerts its influence on the expression of KLF5 and the maintenance of cancer stem cell-like properties by means of downregulating miR-145.

## Introduction

Cervical cancer ranks as the second major gynecological malignancy, with studies suggesting that over half a million women worldwide affected, contributing to an estimated global and annual death toll of more than 300,000 women (1). The greater majority of women affected have been reported to be aged between 20 and 39 years, highlighting the need for improved diagnostic methods for detection among young females (2). Cervical cancer represents a preventable malignancy with a high cure rate if diagnosed during its early stages, that being said, the rate of incidence and mortality remains deeply concerning particularly in the underdeveloped world (3). Cancer stem cells (CSCs) are enriched in side population (SP) cells and possess the capacity to self-renew and differentiate, thus facilitating tumor growth, and enhancing metastatic potential (4). Recently, research into CSCs enriched in cervical cancer has expanded, with the hope of identifying candidate biomarkers with therapeutic benefits for cervical cancer (5).

RETRACTED

Cumulative evidence over the past few years has indicated that non-coding RNAs play a critical role as regulators in a wide array of cancers including cervical cancer, which highlights the urgent need to identify novel biomarkers capable of aiding in the control of disease progression (6). Long non-coding RNAs (lncRNAs) have been suggested to be of potential diagnostic and therapeutic benefit for gynecologic cancers (7). A previous comprehensive analysis of competing endogenous RNA (ceRNA) networks in lung adenocarcinoma identified that LINC00337 may competitively bind to hsa-miR-373 and hsa-miR-519d to mediate their target genes (8). MicroRNAs (miRNAs) represent endogenously expressed small RNAs that have been underlined as either tumor suppressors or oncogenes serving as posttranscriptional mediators of mRNA expression in recent years (9). The abnormal expression of oncogenic or tumor-suppressive miRNAs has been demonstrated to exert a marked influence on cervical carcinogenesis. More specifically, microRNA-145 (miR-145) has been identified as a suppressive factor in the context of cervical cancer cell growth (10). The overexpression of miR-145 could temper cancer stem cell generation as well as the maintenance of cancer stem cell characteristics in cervical cancer cells (11). Interestingly, Kruppel like factor 5 (KLF5) was previously demonstrated as a target gene of miR-145 in the study of Cheng et al. (12). KLF5 has been demonstrated to contribute to the acceleration of the transformation of proliferative phenotype *via* the cyclin D1 promoter (13). Increasing evidence recapped the role of lncRNAs in cervical cancer through regulating miRNAs and mRNAs, and the challenge is now to elucidate the mechanism by which lncRNAs functionally contribute to oncogenic changes. Herein, the current study aimed to identify the effects associated with the LINC00337, miR-145, and KLF5 on the behaviors of CSCs in cervical cancer. We initially isolated sphere-forming cells (SFCs) from HeLa cells. In order to characterize CSCs from SFCs, we evaluated CSC-like features including multi-drug resistance and surface markers of CSCs. The characterization of CD44^+^/CD24^low/−^SFCs made the CSC-like features apparent. We subsequently further demonstrated that LINC00337 is upregulated in CD44^+^/CD24^low/−^SFCs and LINC00337 depletion reduces CSC-like properties of CD44^+^/CD24^low/−^SFCs.

RETRACTED

## Materials and Methods

### Ethics Statement

All animal experiments were performed with the approval from the Institutional Animal Care and Use Committee of The Second Affiliated Hospital of Harbin Medical University.

### Cervical Cancer Cell Lines

Normal cervical epithelial cells (NCECs) and cervical cancer cell lines HeLa, SiHa, CaSki, and C33A (ATCC, USA) were maintained in 10% fetal bovine serum-containing DMEM (Invitrogen, USA).

### Sphere-Forming Assays

HeLa cells were maintained in serum-free DMEM-F12 (Sigma-Aldrich, St. Louis, MO, USA) containing 1 ml of 50 × B27 (Invitrogen, Thermo Fisher Scientific Inc., Waltham, MA, USA), 20 ng/mL human basic fibroblast growth factor (bFGF, Invitrogen) and 20 ng/mL epidermal growth factor (EGF, Invitrogen) utilizing a commercially available a 24-well ultralow attachment plate at 1 × 10^3^ cells per well (Corning Inc., USA). Following a period of 7 days, the SFCs derived from HeLa cells (HeLa-SFCs) were subjected centrifugation (300 × g for 5 min), after which the sphere numbers tallied (14). The spherical cells were treated using a 1:1 diluted 2.5% Trypsin-EDTA (Invitrogen) for 5 min at 37°C followed by passage culture. Next, the spherical cells were separated by means of repeated pipetting, counted, and passed with a cell strainer (40 μm, BD, Brisbane, QLD, Australia). Finally, Hela-SFCs were photographed and counted using an Olympus microscope (Olympus, Tokyo, Japan).

### Fluorescence-Activated Cell Sorting Analysis

The HeLa-SFCs were dispersed into single cell suspensions and stained with antibodies specific for CD44 conjugated with fluorescein isothiocyanate (FITC, Invitrogen) and for CD24 conjugated with Rphycoerythrin (Invitrogen). Immunoreactive HeLa-SFCs were subject to fluorescence-activated cell sorting analysis using an FACSAria III sorter (BD Biosciences, San Jose, CA, USA) in accordance with the manufacturers' instructions, after which the cells exhibiting an expression pattern of CD44^+^/CD24^low/−^ were identified accordingly (15).

### Drug Treatment

The HeLa cells and CD44^+^/CD24^low/−^SFCs were separately cultured in the presence of three clinically used chemotherapy drugs cisplatin (1–2 μg ml^−1^), doxorubicin (0.0625 μg ml^−1^) or epirubicin (0.5 μg ml^−1^) (Sigma-Aldrich) well-known to have a cytotoxic profile for HeLa cells, for a period of 24–72 h, respectively (16).

### Transient Transfection

LINC00337-specific short hairpin RNA (named sh-LINC00337) was designed and delivered into CD44^+^/CD24^low/−^SFCs to specifically blunt LINC00337 using Lipofectamine 2000 reagents (Invitrogen) as per the manufacturer's instructions. Either miR-145 mimic or inhibitor was introduced into CD44^+^/CD24^low/−^SFCs in order to manipulate the expression of miR-145 using Lipofectamine 2000 reagents (Invitrogen) in accordance with the manufacturer's instructions. Cell transfection was performed for a duration of 48 h.

RETRACTED

### RNA Isolation and Quantification

Total RNA extractions by Trizol reagents (Invitrogen) were used to generate cDNA based on the instructions of the PrimeScript RT reagent Kit (Takara, Japan). The relative expressions of targets were quantified using SYBR®Premix Ex TaqTM II (RR820A, Takara Bio Inc., Dalian, China) on the Applied Biosystems 7500 Real-Time PCR System with each reaction run in triplicate (Applied Biosystems, Carlsbad, CA, USA) and subsequently normalized to the expression of GAPDH (for mRNA) and U6 (for miRNA). The primer sequences are listed in Table 1. The delta-delta comparative threshold cycle (ΔΔCt) methods were employed to calculate the fold changes using the formula 2^−ΔΔCT^.

**Table 1:** The primer sequences used for qRT-PCR.

**Target**	**Primer sequence**
LINC00337	F::5′-GGAGATGCACAGAAACACGC-3′
	R::5′-TAGGTGTGTTGTCCCCAAGC-3′
miR-145	F::5′-CAGTCGCCTAGCCAACCCTG-3′
	R: 5′-GCAATG CCGTGGAAGTCAAAT-3′
KLF5	F: 5′-ACCTGGAGAAACGCCGCATC-3′
	R: 5′-AGTGTGAGTCCTCAGGTGAG-3′
MDR-1	F: 5′-CCCATCATTGCAATAGCAGG-3′
	R: 5′-GTTCAAACTTCTGCTCCTGA-3′
Nanog	F: 5′-CAGAAGGCCTCAGCACCTAC-3′
	R: 5′-ATTGTTCCAGGTCTGGTTGC-3′
Sox2	F: 5′-AGCTACAGCATGATGCAGGA-3′
	R: 5′-GGTCATGGAGTTGTACTGCA-3′
Oct4	F: 5′-CAGTGCCCGAAACCCACAC-3′
	R: 5′-GGAGACCCAGCAGCCTCAAA-3′
U6	F: 5′-AACGCTTCACGAATTTGCGT-3′
	R: 5′-CTCGCTTCGGCAGCACA-3′
GAPDH	F: 5′-CTCAACTACATGGTCTACATGTTCCA-3′
	R: 5′-CTTCCCATTCTCAGCCTTGACT-3′

*F, forward; R, reverse*.

### Protein Isolation and Western Blot Analysis

Proteins were extracted using lysis buffer (BIOSS, Beijing, China). Cell lysate proteins were run on 10% SDS-PAGE and then transferred onto polyvinylidene difluoride (PVDF) membranes (Beyotime Institute of Biotechnology). The membranes were probed with primary antibodies to KLF5 (ab137676, 1:100, Abcam, Cambridge, UK), to Sox2 (ab97959, 1:10,000, Abcam), to Oct4 (ab18976, 1:1,000, Abcam), to Nanog (ab21624, 1:200, Abcam), to MDR1 (ab170904, 1: 1,000, Abcam), and to GAPDH (ab8245, 1:10,000, Abcam). Immunoreactive bands were visualized by horseradish peroxidase-labeled goat anti-rabbit IgG and the enhanced chemiluminescence (ECL) reagents.

### Soft-Agar Colony Formation Assays

MEM with 10% FBS and 0.4% agarose was plated in 35 mm diameter plastic dishes as a base layer (1 mL per dish). Single cell suspensions of HeLa-SFCs were mixed with MEM containing 0.7% soft agar. The aforementioned mixture was then overlaid on the base layers. The culture period was performed for 2 weeks, after which the generated colonies were counted under a light microscope (Olympus, Tokyo, Japan).

RETRACTED

### CCK-8 Assays

CD44^+^/CD24^low/−^SFCs were cultured in a 96-well plate, with 10 μl CCK-8 solution (35000, AAT Bioquest, Mercury Drive, Sunnyvale, CA, USA) added to each well at the end of culture (24th, 48th and 72nd h). Each incubation with CCK-8 solution lasted for 4 h. Dimethyl Sulfoxide (150 μL, DMSO, Sigma-Aldrich) was used to dissolve the formazan crystals. Absorbance values were obtained at a wavelength of 450 nm using a Microplate reader (DNM-9602G; Aolu Biotech, Shanghai, China). CCK-8 assays were subsequently performed in order to evaluate the multi-drug resistances of CD44^+^/CD24^low/−^SFCs. In detail, 5 × 10^3^ CD44^+^/CD24^low/−^SFCs were seeded into 96-well plates and incubated with chemotherapeutic drugs cisplatin, doxorubicin and epirubicin (Sigma-Aldrich) for 24–72 h. Four hours later, the plate was incubated with CCK-8 solution at 37°C for 4 h. Absorbance was read at 570 nm using a Microplate reader. The respective concentrations of cisplatin, doxorubicin and epirubicin required to inhibit cell growth by 50% in comparison to vehicle treated control cells (IC50 values) were calculated.

### Cell Cycle and Cell Apoptosis Assays

Cell nuclei were stained with 100 mg/ml of RNase A and 50 mg/ml propidium iodide (PI, Santa Cruz Biotechnology, USA) and then analyzed by flow cytometry (FACScan® BD Biosciences) equipped with CellQuest software (BD Biosciences) to examine the distribution of cells throughout G0/G1, S, and G2/M phases of the cell cycle. For cell apoptosis assays, PI was used in conjunction with Annexin V-FITC (Santa Cruz Biotechnology) as per the manufacturer's instructions to determine if cells were viable, apoptotic, or necrotic by flow cytometry.

### Fluorescence *in situ* Hybridization (FISH)

LncRNA subcellular localization data was obtained from lncatlas.crg.eu. in order to predict the subcellular localization of LINC00337. Next, FISH was performed to further evaluate the subcellular localization of LINC00337 using Ribo^TM^ lncRNA FISH Probe Mix (Red) (Ribo Biotech, Guangzhou, China) as per the manufacturers' instructions. CD44^+^/CD24^low/−^SFCs (6 × 10^4^/well) were mounted onto slides and fixed in 4% formaldehyde. The slides were pretreated by protease K (2 μg/mL), glycine and acetic anhydride, followed by pre-hybridization for 1 h at 42°C. Hybridization was performed overnight at 42°C using probes (250 μL, 300 ng/mL) against LINC00337. Finally, the slides were stained with phosphate-buffered saline with Tween (PBST)-diluted DAPI. Images were acquired using a fluorescence microscope (Olympus, Japan), with five random fields acquired from each slide.

RETRACTED

### Luciferase Assay

The pmirGLO-based luciferase reporter plasmids (Catalog number E1330, Promega, Madisom, WI, USA) containing wild-type LINC00337 (pmirGLO-LINC00337-WT, sense: 5′- GAGCTCCTCTGCGGCCTAGCTTTGT-3′, antisense: 5′- TCTAGAGCACGTTTTCTGAGCACCGT-3′), LINC00337 mutated at the putative miR-145 binding sites (pmirGLO-LINC00337-MUT, sense: 5′- GAGCTCGCCAGGCGAGTGCGGCAGTCTG-3′, antisense: 5′- TCTAGAGCACGTTTTCTGAGCACCGT-3′), wild-type KLF5 (pmirGLO-KLF5-WT, sense: 5′- GAGCTCCCTGGGCTCCCTCAAATGAC-3′, antisense: 5′- TCTAGAGTGCCTGCCAACTGATTTGT-3′), or KLF5 mutated at the putative miR-145 binding sites (pmirGLO-KLF5-MUT, sense: 5′-GAGCTCCAACTAAAACGAAATGTATATTTGAA-3′, antisense: 5′-TCTAGAGTGCCTGCCAACTGATTTGT-3′) were designed. The forward primer contained Sac I sites with the reverse primer contained Xba I sites, all of which were synthesized by GenePharma (Shanghai, China). The HEK293T cells (Shanghai Beinuo Biotech Ltd., Shanghai, China) were seeded into 6-well plates in triplicate and co-transfected with well-designed pmirGLO-based reporter plasmids with either miR-145 mimic or mimic control using the dual-luciferase reporter assay system based on the manufacturer's instructions (D0010, Beijing Solarbio Science & Technology Co., Ltd, China). The relative luciferase activity was normalized to that of Firefly luciferase.

### RNA-Biotin Pull-Down Assays

CD44^+^/CD24^low/−^SFCs were treated with wild-type or mutated miR-145 labeled by the Biotin RNA Labeling Mix (Roche Applied Sciences, Indianapolis, IN, USA), with incubation in lysis (Ambion, Austin, Texas, USA) performed 48 h later for 10 min. The cell lysates were treated with RNase-free DNase I (Sigma-Aldrich Chemical Company, St Louis, MO, USA) and incubated with streptavidin coated magnetic beads (Sigma-Aldrich Chemical Company) at 4°C for 3 h. RNA was subsequently extracted from the complexes for qRT-PCR analyses purposes.

### RNA Immunoprecipitation (RIP)

CD44^+^/CD24^low/−^SFCs were lysed in RIP Lysis Buffer at 4°C for 30 min. Cell extracts were incubated with protein A/G sepharose beads conjugated with antibodies against Ago2 (P10502500, Otwo Biotech, Shenzhen, China) or normal mouse IgG. Immunoprecipitated RNA and total RNA from the whole cell lysates (input controls) were extracted for qRT-PCR analyses.

### Cervical Cancer Xenograft Animal Models

Non-obese diabetic, severe combined immunodeficient (NOD/SICD) mice (17) (without limitation in gender, aged 4–6 weeks, weighing 18–25 g) were purchased from Guangdong Medical Laboratory Animal Center (Guangdong, China). The mice were initially subcutaneously injected (1 × 10^6^ cells per mouse) with CD44^+^/CD24^low/−^SFCs with either lentiviral particles harboring sh-LINC00337 or scramble shRNA. All the aforementioned lentiviral vectors were purchased from Dharmacon Company (Lafayette, CO, USA). The growth of human cervical cancer xenografts was monitored at 7, 14, 21, and 28 days following implantation. The mice were euthanized by means of cervical dislocation at 28 days.

RETRACTED

### Statistical Analysis

All statistical analyses were reflective of three independent experiments (each in triplicate) and conducted using SPSS 21.0 software (IBM, Armonk, NY, USA), with two-tailed *p* < 0.05 as a level of statistical significance. For statistical comparisons, independent-sample *t*-test, a one-way analysis of variance (ANOVA) with Tukey's test, and repeated measurements ANOVA with Bonferroni test were performed as required.

## Results

### The Expression Patterns of LINC00337 in Cervical Cancer and Phenotypic Characterization of HeLa-SFCs

We initially analyzed the expression of LINC00337 in cervical cancer samples as well as the adjacent normal samples from the TCGA database. As depicted in Figure 1A (*p* < 0.01), LINC00337 was upregulated in cervical cancer tissues. Next, to further assess the expression pattern of LINC00337 in cervical cancer, we quantified LINC00337 in NCECs and cervical cancer cell lines HeLa, SiHa, CaSki and C33A by means of qRT-PCR analysis. The results obtained indicated that the relative expression of LINC00337 was notably higher in HeLa, CaSki, and C33A cells than in NCECs, while the HeLa cells were identified to have exhibited the greatest fold changes in LINC00337 among the cervical cancer cells (*p* < 0.05, Figure 1B). Fluorescence-activated cell sorting analysis was performed to detect the phenotypic characterization of HeLa-SFCs using surface markers of CD44 and CD24. The results demonstrated that HeLa-SFCs were highly enriched (85 ± 6%) in CD44(high)CD24(negative) subpopulations (Figure 1C). Next, investigation into whether CD44^+^/CD24^low/−^SFCs exhibited CSC-like features was conducted. We subsequently cultured CD44^+^/CD24^low/−^SFCs in the sphere culture conditions containing chemotherapy drugs (cisplatin, doxorubicin, or epirubicin) and detected their sphere-formation abilities to test the resistance of CD44^+^/CD24^low/−^SFCs to multi-drug resistant. As illustrated in Figure 1D, CD44^+^/CD24^low/−^SFCs cultured in the presence of cisplatin, doxorubicin, and epirubicin displayed no significant difference in regard to the sphere-formation abilities when compared with parental HeLa cells cultured in sphere culture medium without chemotherapy drugs. Afterwards, we determined Sox2, Nanog, and Oct4 all of which represent core stem cell transcription factors, associated with the pluripotency of CSCs. The qRT-PCR analysis and western blot analysis results demonstrated that the expression of Nanog, Sox2, and Oct4 in CD44^+^/CD24^low/−^SFCs were higher than those in non-CD44^+^/CD24^low/−^SFCs (*p* < 0.05, Figures 1E,F). Additionally, we quantified LINC00337 in HeLa-SFCs and identified that the relative expression of LINC00337 was higher in CD44^+^/CD24^low/−^SFCs than in that of the non-CD44^+^/CD24^low/−^SFCs (*p* < 0.05, Figure 1G). These findings provided evidence verifying that CD44^+^/CD24^low/−^SFCs exhibit CSC-like traits and LINC00337 which warranted further investigated as a critical governor of cancer stem cell generation and the maintenance of cancer stem cell characteristics in cervical cancer cells.

RETRACTED

**Figure 1:** Expression pattern of LINC00337 in cervical cancer and phenotypic characterization of HeLa-SFCs. **(A)** The expression pattern of LINC00337 in cervical cancer samples (*n* = 306) and adjacent normal samples (*n* = 13) from TCGA database. **(B)** LINC00337 expression was quantified in NCECs and cervical cancer cell lines HeLa, SiHa, CaSki, and C33A using the qRT-PCR analysis, normalized to GAPDH expression; data are shown as mean ± standard deviation of three technical replicates and analyzed by one-way ANOVA (*p < 0.05 vs. NCECs). **(C)** Identification of CD44^+^/CD24^low/−^SFCs by fluorescence-activated cell sorting analysis; **(D)** Multi-drug resistance of CD44^+^/CD24^low/−^SFCs; CD44^+^/CD24^low/−^SFCs were maintained in sphere culture medium separately supplemented with working concentrations of cisplatin, doxorubicin and epirubicin, compared with parental HeLa cells cultured in sphere culture medium without these drugs (×40). **(E)** The mRNA expression of Nanog, Sox2, and Oct4 in CD44^+^/CD24^low/−^SFCs and non-CD44^+^/CD24^low/−^SFCs were determined by the qRT-PCR analysis, normalized to GAPDH expression. **(F)** Representative Western blots of Nanog, Sox2 and Oct4 in CD44^+^/CD24^low/−^SFCs and non-CD44^+^/CD24^low/−^SFCs and their quantitative analyses. **(G)** LINC00337 expression was quantified in CD44^+^/CD24^low/−^SFCs and non-CD44^+^/CD24^low/−^SFCs using the qRT-PCR analysis, normalized to GAPDH expression; data are shown as mean ± standard deviation of three technical replicates and analyzed by non-paired *t*-test (*p < 0.05 *vs*. non-CD44^+^/CD24lo^w/−^SFCs).

### LINC00337 Knockdown Impairs the Maintenance of CSC-Like Properties of CD44^+^/CD24^low/-^SFCs

Since CD44^+^/CD24^low/−^SFCs exhibited the characteristics of CSCs, we subsequently set out to investigate the biological function of LINC00337 in CD44^+^/CD24^low/−^SFCs. We synthesized a shRNA to silence the expression of LINC00337, and 48 h later knockdown of LINC00337 by 85% in CD44^+^/CD24^low/−^SFCs relative to scramble shRNA-treated CD44^+^/CD24^low/−^SFCs was achieved (*p* < 0.05, Figure 2A). Forty-eight hours after sh-LINC00337 or scramble shRNA treatment to CD44^+^/CD24^low/−^SFCs, sphere-forming assays and soft-agar colony formation assays were performed, the results of which demonstrated that LINC00337 knockdown diminished colonies in soft-agar and generation of tumorospheres in CD44^+^/CD24^low/−^SFCs (*p* < 0.05, Figures 2B,C). The CCK-8 assay results illustrated that LINC00337 knockdown decreased cell viability (*p* < 0.05, Figure 2D) and reduced IC50 values of cisplatin, doxorubicin and epirubicin in CD44^+^/CD24^low/−^SFCs (*p* < 0.05, Figure 2E). The flow cytometric analysis revealed more CD44^+^/CD24^low/−^SFCs arrested in the G0/G1 phase (Figure 2F) and more apoptotic CD44^+^/CD24^low/−^SFCs (Figure 2G) upon LINC00337 knockdown. The qRT-PCR analysis and western blot analysis findings demonstrated that the expressions of multi-drug resistance gene-1 (MDR-1), Nanog, Sox2, and Oct4 in the LINC00337-depleted CD44^+^/CD24^low/−^SFCs were decreased more so than those in the scramble shRNA-treated CD44^+^/CD24^low/−^SFCs (*p* < 0.05, Figures 2H,I). The aforementioned findings suggested that LINC00337 knockdown suppressed self-renewal abilities while promoting the apoptosis of the CSCs in cervical cancer.

RETRACTED

**Figure 2:** LINC00337 knockdown prevents CSC-like properties of CD44^+^/CD24^low/−^SFCs. **(A)** CD44^+^/CD24^low/−^SFCs were transfected with sh-LINC00337 or scramble shRNA for 48 h. 85% knockdown of LINC00337 in CD44^+^/CD24^low/−^SFCs was validated by the qRT-PCR analysis. **(B)** Statics of spheres per 1,000 cells upon LINC00337 knockdown. **(C)** Views and numbers of colonies in CD44^+^/CD24^low/−^SFCs upon LINC00337 knockdown, examined by soft-agar colony formation assays. **(D)** CCK-8 assays were performed to evaluate the viability of CD44^+^/CD24^low/−^SFCs upon LINC00337 knockdown. **(E)** IC50 values of cisplatin, doxorubicin and epirubicin in CD44^+^/CD24^low/−^SFCs upon LINC00337 knockdown. **(F)** Cell cycle distribution of CD44^+^/CD24^low/−^SFCs was determined by flow cytometric analysis of PI staining upon LINC00337 knockdown. **(G)** Cell apoptosis of CD44^+^/CD24^low/−^SFCs was determined by flow cytometric analysis of Annexin V-FITC/PI double staining upon LINC00337 knockdown. **(H)** The mRNA expressions of MDR-1, Nanog, Sox2, and Oct4 in CD44^+^/CD24^low/−^SFCs were determined by the qRT-PCR analysis upon LINC00337 knockdown. **(I)** Representative Western blots of MDR-1, Nanog, Sox2, and Oct4 and their quantitative analyses in CD44^+^/CD24^low/−^SFCs upon LINC00337 knockdown. Data are shown as mean ± standard deviation of three technical replicates and analyzed by non-paired *t*-test and by two-way ANOVA (only for panel **D**); *p < 0.05 and **p < 0.01 vs. scramble shRNA.

RETRACTED

### LINC00337 Is Cytoplasm-Sub-Localized in CD44^+^/CD24^low/-^SFCs

Emerging evidence supports the ceRNA hypothesis that implicated in the carcinogenesis of cervical cancer (18). We speculated that LINC00337 may function as a ceRNA participate in carcinogenesis of cervical cancer. We initially explored the LncATLAS database for the subcellular localization of LINC00337 with the database revealed that LINC00337 is cytoplasm-sublocalized (Figure 3A). Subsequent FISH experiments with probes targeting LINC00337 were performed in an attempt to validate the subcellular localization of LINC00337 in the CD44^+^/CD24^low/−^SFCs. As depicted in Figure 3B, the CD44^+^/CD24^low/−^SFCs were stained with probes targeting LINC00337 (red stain), and the nuclei were stained with DAPI (blue stain). The merged image illustrated that LINC00337 was cytoplasm-sublocalized in the CD44^+^/CD24^low/−^SFCs.

**Figure 3:** Subcellular localization of LINC00337 in CD44^+^/CD24^low/−^SFCs. **(A)** Subcellular localization of LINC00337 documented in the LncATLAS database. **(B)** FISH experiments with probes targeting LINC00337 were performed to validate the subcellular localization of LINC00337 in CD44^+^/CD24^low/−^SFCs; CD44^+^/CD24^low/−^SFCs were stained with probes targeting LINC00337 (red stain), and the nuclei were stained with DAPI (blue stain). The merged image showed LINC00337 was cytoplasm-sublocalized in CD44^+^/CD24^low/−^SFCs. Original magnification, × 400.

### LINC00337 Regulates KLF5 Expression by Competing for miR-145 in CD44^+^/CD24^low/-^SFCs

Next, the emphasis of the *in vitro* experiments was geared toward an investigation into the mechanism associated with LINC00337 and the regulation of CSCs in cervical cancer. In order to determine whether LINC00337 regulates target genes using a similar mechanism, we initially performed a computer-based lncRNA-miRNA-mRNA target detection programs (https://cm.jefferson.edu/rna22/Interactive/) highlighting the binding sites of miR-145 in the 3′-UTR of LINC00337 and KLF5 (Figure 4A). Next, to ascertain as to whether both LINC00337 and KLF5 could bind to miR-145, dual-luciferase reporter gene assays were conducted. Diminished luciferase activity at vectors containing the LINC00337 and KLF5 3′-UTR with recognizing sites in the presence of miRNA-451 mimic were detected (*p* < 0.05, Figure 4B). Next, LINC00337 was assessed in order to determine whether it could bind to miR-145 and function as a ceRNA. As expected, a greater degree of LINC00337 enrichment was identified by the RNA pull-down assays followed by qRT-PCR analysis (*p* < 0.05, Figure 4C). LINC00337-Ago2 immunoprecipitation was performed in the CD44^+^/CD24^low/−^SFCs treated with miR-145 inhibitor. RIP-qPCR assay results indicated that LINC00337 or miR-145 immunoprecipitation by anti-ago2 were elevated relative to anti-IgG (*p* < 0.05, Figure 4D). The qRT-PCR analysis and western blot analysis findings revealed upregulated miR-145 and downregulated KLF5 in CD44^+^/CD24^low/−^SFCs following LINC00337 knockdown. We subsequently performed gain- and loss-of function studies in CD44^+^/CD24^low/−^SFCs in order to validate the regulation of miR-145 on KLF5. As expected, our results revealed that miR-145 promotion by its specific mimic inhibited the expression of KLF5. Additionally, miR-145 inhibition by its specific inhibitor increased the activity of KLF5 in CD44^+^/CD24^low/−^SFCs, whereas subsequent LINC00337 knockdown decreased the expression of KLF5 in the CD44^+^/CD24^low/−^SFCs (*p* < 0.05, Figures 4E,F). Taken together, the data obtained revealed that LINC00337 could function as a ceRNA and positively regulate KLF5 by means of sponging miR-145 in CD44^+^/CD24^low/−^SFCs.

RETRACTED

**Figure 4:** LINC00337 functions as a ceRNA of miR-145 and positively regulates KLF5 in CD44^+^/CD24^low/−^SFCs. **(A)** Putative miR-145 binding sites on the LINC00337 promoter and the KLF5 mRNA 3′UTR by computer-based lncRNA-miRNA-mRNA target detections (https://cm.jefferson.edu/rna22/Interactive/). **(B)** The luciferase activity of reporter vectors containing the LINC00337 promoter or HMGB1 3′-UTR with recognizing sites or recognizing sites mutated in the presence of miR-145 mimic; **p < 0.01 vs. miR-NC. **(C)** LINC00337 precipitation pulled down by biotinylated wild-type (miR-145-Bio) or mutated (miR-145-MUT-Bio) miR-145 sequence by RNA pull-down assays and the qRT-PCR analysis, relative to mock probes (NC-Bio); **p < 0.01 vs. NC-Bio. **(D)** LINC00337 or miR-145 immunoprecipitated by anti-Ago2 antibody was determined by RIP-qPCR assay, relative to anti-IgG antibody; **p < 0.01 vs. anti-IgG. In the following experiments, CD44^+^/CD24^low/−^SFCs were transfected with sh-LINC00337, scramble shRNA, miR-145 mimic, mimic control, miR-145 inhibitor, inhibitor control, and shRNA-LINC00337 plus miR-145 inhibitor for 48 h. **(E)** The expression of miR-145 (normalized to U6 expression) and the mRNA expression of KLF5 (normalized to GAPDH expression) were determined by the qRT-PCR analysis; **p < 0.01 vs. corresponding controls. **(F)** Representative Western blot of KLF5 and its quantitative analysis, normalized to GAPDH expression; **p < 0.01 *vs*. corresponding controls. Data are shown as mean ± standard deviation of three technical replicates and analyzed by one-way ANOVA.

RETRACTED

### LINC00337 Regulates CSC-Like Properties of CD44^+^/CD24^low/-^SFCs *via* miR-145

Next, we aimed to determine whether miR-145-dependent KLF5 participated in the regulatory mechanism associated with LINC00337 in CD44^+^/CD24^low/−^SFCs. Forty 8 h after cell treatment, sphere-forming assays and soft-agar colony formation assays illustrated the restoration of miR-145 using mimic yield results of reduced sphere formations and colonies, while disruption of miR-145 using an inhibitor resulted in a greater amount of sphere formations and colonies compared with mimic or inhibitor control, respectively (*p* < 0.05, Figures 5A,B). The subsequent CCK-8 assays results revealed that the miR-145 mimic reduced cell viability along with IC50 values of cisplatin, doxorubicin and epirubicin, while the miR-145 inhibitor produced a contrasting trend with opposite results (*p* < 0.05, Figures 5C,D). The flow cytometric analysis revealed fewer CD44^+^/CD24^low/−^SFCs arrested in the G0/G1 phase (Figure 5E) and fewer apoptotic CD44^+^/CD24^low/−^SFCs (Figure 5F) upon miR-145 elevation. The miR-145 inhibitor likewise produced a contrasting trend with opposite results The qRT-PCR analysis and western blot analysis displayed a decrease in the expressions of MDR-1, Nanog, Sox2, and Oct4 in CD44^+^/CD24^low/−^SFCs with elevated expression of miR-145 (*p* < 0.05, Figures 5G,H). In contrast, miR-145 inhibitor increased expressions of Nanog, Sox2 and Oct4 in CD44^+^/CD24^low/−^SFCs. Results also revealed loss of function of miR-145 inhibitor on the sphere formations, colonies, cell viability, IC50 values, cell cycle progression, cell apoptosis, and expressions of MDR-1, Nanog, Sox2 and Oct4upon LINC00337 knockdown. Altogether, the aforementioned results support the notion that LINC00337 regulates CSC-like properties of CD44+/CD24^low/−^SFCs *via* miR-145.

**Figure 5:** LINC00337 regulates CSC-like properties of CD44^+^/CD24^low/−^SFCs *via* miR-145. CD44^+^/CD24^low/−^SFCs were transfected with miR-145 mimic, mimic control, miR-145 inhibitor, inhibitor control, sh-LINC00337 plus miR-145 inhibitor, and scramble shRNA plus inhibitor control for 48 h. **(A)** Statics of spheres per 1,000 cells. **(B)** Views and numbers of colonies in CD44^+^/CD24^low/−^SFCs, examined by soft-agar colony formation assays. **(C)** CCK-8 assays were performed to evaluate the viability of CD44^+^/CD24^low/−^SFCs. **(D)** IC50 values of cisplatin, doxorubicin and epirubicin in CD44^+^/CD24^low/−^SFCs. **(E)** Cell cycle distribution of CD44^+^/CD24^low/−^SFCs was determined by flow cytometric analysis of PI staining. **(F)** Cell apoptosis of CD44^+^/CD24^low/−^SFCs was determined by flow cytometric analysis of Annexin V-FITC/PI double staining. **(G)** The mRNA expressions of MDR-1, Nanog, Sox2, and Oct4 in CD44^+^/CD24^low/−^SFCs were determined by the qRT-PCR analysis, normalized to GAPDH expression. **(H)** Representative Western blots of MDR-1, Nanog, Sox2, and Oct4 and their quantitative analyses in CD44^+^/CD24^low/−^SFCs, normalized to GAPDH expression. Data are shown as mean ± standard deviation of three technical replicates and analyzed by one-way ANOVA, for **(C)**, by two-way ANOVA for **(C)**. *p < 0.05 vs. mimic control. **p < 0.01 vs. mimic control. ^#^*p* < 0.05 vs. inhibitor control. ^*##*^*p* < 0.01 vs. inhibitor control.

RETRACTED

### LINC00337 Knockdown Attenuates Tumorigenicity of CD44^+^/CD24^low/-^SFCs

As previously mentioned, our results identified that LINC00337 knockdown could reduce CSC-like properties of CD44^+^/CD24^low/−^SFCs *in vitro*. In order to further verify that the *in vivo* results could be reproduced in *in vivo* studies, we subcutaneously injected CD44^+^/CD24^low/−^SFCs with either lentiviral particles containing sh-LINC00337 or scramble shRNA into NOD/SCID mice. As expected, the results demonstrated that the LINC00337 knockdown triggered reductions in tumor volume and weight in mice (*p* < 0.05, Figures 6A–C), ultimately suggesting that LINC00337 knockdown reduces tumorigenicity of CD44^+^/CD24^low/−^SFCs. We next determined an elevation in miR-145 expression with a decline in KLF5 expression in tissue sections of xenografted tumors upon LINC00337 knockdown by RT-qPCR (Figure 6D).

**Figure 6:** LINC00337 knockdown attenuates tumorigenicity of CD44^+^/CD24^low/−^SFCs. NOD/SICD mice were subcutaneously injected with CD44^+^/CD24^low/−^SFCs with either lentiviral particles containing shRNA-LINC00337 (*n* = 9) or scramble shRNA (*n* = 9) at 1 × 10^6^ cells per mouse. Twenty-eight days later, the mice were euthanized by cervical dislocation. **(A)** The tumor growth curves at the 7th, 14th, 21st, and 28th day after subcutaneous injection of CD44^+^/CD24^low/−^SFCs; Data are shown as mean ± standard deviation of three technical replicates and analyzed by two-way ANOVA. **(B)** Representative views of tumors 28 days after subcutaneous injection of CD44^+^/CD24^low/−^SFCs. **(C)** The tumor weight of mice 28 days after subcutaneous injection of CD44^+^/CD24^low/−^SFCs. **(D)** The expression of miR-145 and KLF-5 in tissue sections of xenografted tumors upon LINC00337 knockdown was determined by RT-qPCR. Data are shown as mean ± standard deviation of three technical replicates and analyzed by non-paired *t*-test. *p < 0.05 vs. scramble shRNA. **p < 0.01 *vs*. scramble shRNA.

RETRACTED

## Discussion

Accumulating evidence continues to lend support to the notion that CSCs are enriched in tumor cells and possess a strong ability to self-renew and differentiate into tumor cells, which can ultimately facilitate tumor growth and enhance metastatic potential (4). The silencing of oncogenes in cervical CSCs have been speculated to temper their growth as well as the sphere formation *via* regulating the self-renewal pathway. Notably, numerous studies have provided evidence regarding the roles of lncRNAs in the regulation of cell behaviors in cervical cancer through the lncRNA-miRNA-mRNA interaction (19, 20). Herein, our study aimed to investigate the regulation of the LINC00337, miR-145, and KLF5 from a cervical cancer perspective. Overall, our findings suggest that LINC00337 knockdown leads to KLF5 inhibition and impairs the maintenance of CSC-like properties of CD44^+^/CD24^low/−^SFCs by regulating miR-145.

LncRNAs have displayed potential significant implications from a diagnostic as well as a prognostic point of view in the form of biomarkers in cervical cancer. A previous report concluded that the upregulated expression pattern of lncRNA PVT1 is associated with poor prognosis (21). A key observation made during our study indicated that LINC00337 was highly expressed in cervical cancer. Downregulated LINC00337 diminished the capability of cervical CSCs to form colonies in soft-agar and generate tumorospheres, while stunting the self-renewal and promoting the apoptosis of cervical CSCs. A recent study demonstrated a ceRNA network related to LINC00337 in esophageal squamous cell carcinoma. A recent study demonstrated a ceRNA network related to LINC00337 in esophageal squamous cell carcinoma (22). LINC00337 may assume the role of a ceRNA to decay hsa-miR-373 and hsa-miR-519d, thus modulating their downstream target genes in lung adenocarcinoma from previous evidence (8). Certain studies have suggested the oncogenic role of lncRNAs in CSCs. The downregulation of lncRNA HOTAIR has been previously reported to impair the retention of colorectal CSCs, highlighting its role as a tumor suppressor (23). Moreover, the lncRNA XIST/miR-200c axis mediates the stemness properties and tumorigenicity of bladder CSC-like cells while the knockdown of XIST possesses the capacity to decrease colony formation as well as the self-renewal ability of miR-200c (24).

Growing evidence has emphasized the significant modulation of lncRNAs and miRNAs in wide range of biological processes of cancer cells by their regulation on mRNAs in human cancers including cervical cancer (25). LINC00337 has been shown to sponge miR-145 to inhibit its regulation on targets. LncRNAs has been reported to bind to miRNAs as ceRNAs and subsequently upregulate the target mRNAs of miRNAs in an indirect manner (26). For example, the lncRNA LINC01116 has been reported in previous research studies to impede tumor progression by decaying miR-145 and upregulating ESR1 in breast cancer (27). Likewise, in the current study, we identified that LINC00337 could bind to miR-145 that targets and negatively regulates KLF5 gene. Consistent with the findings of the current study, the binding sites of miR-145 in the 3′UTR of KLF5 mRNA has also been highlighted in existing literature, and this event has been shown to regulate vascular neointimal lesion formation by means of modulating smooth muscle cell phenotypes (12). Furthermore, KLF5 was shown to be upregulated by lncRNA PVT1 and enhance the tumorigenesis of triple-negative breast cancer *in vivo* (28). Hence, we set out to elucidate the involvement of the LINC00337, miR-145, and KLF5 in the process of mediating the self-renewal of cervical CSCs.

RETRACTED

Importantly, upregulated miR-145 was observed to negate the contributory role of LINC00337 in sustaining cervical CSCs. Wei *et al*. provided evidence suggesting that miR-145 is poorly expressed in the setting of cervical cancer with the potential to serve as a candidate biomarker for detecting cervical cancer and an indicator for predicting the efficacy of radiosensitivity (29). Reduced miR-145 expression has been linked with advanced stages and poor differentiation and its restoration could sensitize cervical cancer to irradiation *in vitro* and *in vivo* by targeted inhibition of HLTF (30). Furthermore, lncRNA MALAT1 silencing has been shown to deteriorate cervical cancer cell colony formation ability while acting to facilitate apoptosis by means of up-regulating the expression of miR-145 (31). Interestingly, KLF5 acts as a candidate biomarker for cervical cancer (32). Functionally, KLF5 facilitates tumor cell proliferation and invasiveness *in vitro* and tumorigenicity and liver metastasis *in vivo* in cervical squamous cell carcinoma (33). It is reasonable to conclude that LINC00337 knockdown impairs the maintenance of CSC-like properties of CD44^+^/CD24^low/−^SFCs by decaying miR-145 and downregulating KLF5.

In conclusion, the key observations of the current study provide evidence pertaining to the implication of the LINC00337, miR-145, and KLF5 in cervical cancer, particularly in mediating the maintenance of CSC-like properties of CD44^+^/CD24^low/−^SFCs in cervical cancer cells. Our findings provide an enhanced understanding of mechanism underlying the aggressive behavior of cervical cancer (summarized in Figure 7). Silencing of LINC00337 was found to attenuate the development of cervical cancer by means of impairing the miR-145-dependent inhibition of KLF5. Considering drug sensitization is associated with the acquisition and maintenance of CSCs in cervical cancer, we will set out to ascertain the effects of LINC00337 knockdown more specifically on drug sensitization and the molecular mechanism responsible for drug sensitization in cervical cancer in our future study. Additionally, the conclusion that LINC00337 maintains stem-cell like traits of cervical cancer cells by regulating miR-145 and KLF5 should be further confirmed by performing a series of experiments in the setting of KLF5 knockdown as well as invasion/metastasis assays under *in vivo* setting.

RETRACTED

**Figure 7:** A systematic diagram depicting the specific mechanism of the LINC00337/miR-145/KLF5 axis in regulating the acquisition and maintenance of cervical cancer stem cells. LINC00337 functions as a ceRNA, positively regulates KLF5 by means of sponging miR-145, and mediates the stem-cell like traits of cervical cancer cells.

## Data Availability Statement

The raw data supporting the conclusions of this article will be made available by the authors, without undue reservation.

## Ethics Statement

The animal study was reviewed and approved by the Institutional Animal Care and Use Committee of The Second Affiliated Hospital of Harbin Medical University.

## Author Contributions

QH was responsible for study design and manuscript editing. WW for data acquisition and data analysis. YC for literature research and manuscript preparation. All authors have reviewed and approved the final submitted manuscript. All authors contributed to the article and approved the submitted version.

## Conflict of Interest

The authors declare that the research was conducted in the absence of any commercial or financial relationships that could be construed as a potential conflict of interest.
